# The Progress of Social Isolation in Patients with Enterostomy during Discharge Transition Period

**DOI:** 10.1155/2022/4940946

**Published:** 2022-07-04

**Authors:** Heqian Ji, Yaru Zhu, Yinuo Wang, Aimin Wang

**Affiliations:** School of Nursing, Qingdao University, Qingdao 266071, China

## Abstract

In terms of social and psychological health of enterostomy patients during hospitalization and discharge transition period, the degree of social isolation in patients during discharge transition period is higher than that during hospitalization period, which is usually manifested by poor self-perception of body image changes. Self-esteem (shame) frustration, severe negative emotions, low psychosocial adjustment, and other factors are closely related to postoperative complications, coping self-efficacy, social support level, family living conditions, and other influencing factors. This is an important reason why patients are difficult to adapt to ostomy life and low quality of life. At present, it is believed that the social isolation related evaluation scale can be used to understand the status quo of patients with social isolation and provide nursing guidance, so as to better cope with the adverse medical outcomes caused by social isolation.

## 1. Introduction

Enterostomy is an operation that connects the intestinal lumen with the abdominal wall. It can be divided into preventive enterostomy and permanent enterostomy according to whether the anus is preserved or not [1]. The incidence of postoperative complications related to stomostomy is as high as 81.1% [2], seriously affecting the physical and mental health of patients. In terms of the psychosocial health of enterostomy patients during hospitalization and discharge transition period, multiple evidences show that the degree of social isolation of patients during discharge transition period is higher than that during hospitalization, which is usually manifested as poor body image change, poor self-perception, frustrated self-esteem (stigma), severe negative emotions, and low psychosocial adaptation [3]. It is closely related to postoperative complications, coping self-efficacy, social support level, family living situation, and other influencing factors [4, 5] and is an important reason for patients' difficulty in adapting to ostomy life and low quality of life [6, 7]. Currently, it is believed that the use of social isolation related assessment scale can understand the status of patients' social isolation and provide nursing guidance [8], so as to better cope with the adverse medical outcomes caused by social isolation. However, at present, few studies have discussed the social isolation of patients with preventive and permanent enterostomy during discharge transition period, which has limited the research progress. Therefore, this review is as follows.

## 2. The Concept of Social Isolation and Its Development

Social isolation is also known as social isolation, and there is no evidence to prove its earliest origin. The word “social isolation” first appeared in the book introduction to Sociology coauthored by Parker and Puji. It refers to voluntary or involuntary collective social activities aimed at social goals. The other theory of social isolation was first proposed by Berkman and Syme [9] in 1965, when they studied the relationship between social networks and death and accidentally found that the older people without social connections were more prone to death, which has been recognized by most scholars. At present, the concept of social isolation is still being improved, which can be summed up as a state of active or passive social derailment that induces negative physiological and psychological results [10].

In the 9 years since the publication of Berkman's theory, social isolation has gradually become an effective predictor of health status and mortality risk. Kaplan and Camacho [11] first proposed that death events induced by poor self-perceived health level have nothing to do with social isolation. Subsequently, Haan et al. [12] also included social isolation as one of the evaluation criteria when studying the correlation between socioeconomic status difference and health status. Seeman et al. [13], such as the social relations in accordance with the present situation of marriage and the relationship with friends and family, church relationship and other social groups can be divided into four dimensions, found complete marriage, good relationships with family and friends are under the age of 60, the protection of the subjects aged 60 and above factors, the prompt social isolation as health evaluation index of high application value.

In 1988, House et al. [14] took the lead in publishing a landmark epidemiological literature review study, which summarized the harms brought by social isolation for the first time, including inducing suicide, increasing the risk of accidents, and increasing the risk of diseases (tuberculosis, schizophrenia, etc.), which attracted wide attention abroad [15]. With the development of medical science and technology, enterostomy has become an important treatment method for colorectal cancer. Evaluation of social isolation of patients with preventive and permanent enterostomy during the transition period of discharge from hospital and providing nursing guidance may help fill in the research gap of social isolation in China [15].

## 3. The Assessment Tools for Social Isolation in Enterostomy Patients during Discharge Transition

### 3.1. The Assessment of Readiness for Hospital Discharge Scale (RHDS)

The readiness for hospital discharge scale is an important indicator to measure whether patients have the ability to discharge and further recover during the discharge transition period. It is closely related to the degree of disease progression and incidence of adverse medical events. It is of great significance to evaluate patients' discharge readiness in order to establish the safety guarantee for patients' transition from discharge to family and society [16].

Weiss and Piacentine [17] prepared RHDS in 2006 on the basis of Perceived Readiness for Discharge After Birth Scale (PRDBS) [18], changing the nature of the scale from specialized to universal. Therefore, it is suitable for patients with enterostomy. The scale consists of four dimensions (personal status, disease knowledge, coping ability, and expected support) and 23 items. The 22 items except the first item are summed up according to 10-point Likert scale. The final total score is positively proportional to the patient's discharge readiness, that is, the higher the score, the better the discharge readiness [19]. It has been proved that the Cronbach's *α* coefficient and content validity of the Sinicized RHDS are 0.97 and 0.97, respectively [20], indicating that the scale has good reliability and validity. Zhou and Yan [21] conducted RHDS investigation on 202 patients with preventive and permanent enterostomy, and the results showed that the patients' overall discharge preparation was poor, which was related to patients' occupation, medical security, and other influencing factors, and played an important role in preventing social isolation of patients, providing a new idea for nursing management of medical staff.

### 3.2. The Assessment of Stigma

The process of stigma assessment is shown in Figure 1.

#### 3.2.1. Social Impact Scale (SIS)

According to reports [22], there are about 100,000 new permanent colostomy patients in China every year, and patients are often accompanied by strong stigma due to changes in body image and other reasons, which seriously affects the prognosis of patients. Regular follow-up of patients' stigma with SIS for a period of time after discharge can help to understand their progress in social isolation.

SIS was compiled by Fife and Wright [23] in 2000. It was used to assess stigma in AIDS or cancer patients. It was proved to be a negative influence in various diseases. In 2007, it was applied to the measurement of stigma of patients with depression after the Han nationality scholar Pan [24] and other Han dynasties. The scale contained four dimensions and 24 items, namely, social exclusion (9 items) and social isolation (7 items). The Fife [23] was used to assess the stigma of patients with depression. Internalized stigma (5 items) and no economic security (3 items), using Likert 4-point scoring method to add points for summation, the higher the patient's self-assessment score, the stronger the sense of stigma. Shen [22] and others used the simplified Chinese version of SIS to evaluate the stigma of 200 patients with permanent enterostomy, reduced the items of the scale to 20, and found Cronbach's of the scale *α*. The coefficient is 0.916, Cronbach's of four dimensions *α*. The coefficient ranged from 0.708 to 0.835, and the test-retest reliability was 0.872. And the fitting indexes of the confirmatory factors of the scale fit well. It has excellent application in avoiding the social isolation of patients with enterostomy and is worth popularizing. Gao et al. [25] measured 193 hospitalized patients with permanent and preventive enterostomy with Chinese version SIS to evaluate the sense of shame and found that patients with permanent enterostomy had higher scores of sense of shame. Ye et al. [4] assessed the stigma of 220 patients with prophylactic enterostomy within 5 months after discharge and found that the patients had a high score of stigma during the discharge transition period. The patients could have self-isolation behavior due to fear that the stoma could not be returned, and the sense of social isolation was aggravated, which should be paid high attention.

#### 3.2.2. Perceived Social Support Scale (PSSS)

Research shows [26] that the degree of social support is closely related to the level of stigma, self-esteem, and expectation of enterostomy patients. Low degree of social support can easily lead to psychological problems such as stigma, frustrated self-esteem, and poor level of hope, which is an important reason for the social isolation of patients. PSSS was used to evaluate patients' sense of social isolation in order to improve their condition and prevent deaths.

PSSS was developed by Zimet et al. [26] in 1987. The scale consists of 3 dimensions (family support, friends support, and other people support) and 24 items. The 5-point Likert scoring method was adopted to add and sum, and it was initially used to evaluate the level of social support felt by college students. The Cronbach's *α* coefficients of the total scale and the three dimensions were 0.88, 0.91, 0.87, and 0.85, respectively, indicating that the scale had high reliability and validity. A few years later, Ye et al. revised the PSSS, reducing the measurement items to 12 and using 7-point Likert scoring method, which has been applied in cancer patients [4]. Comrade [27], such as a random sample of 106 patients with permanent colostomy mouth line 1 ~ 12 months follow-up not long out of the hospital at the same time, the use of PSSS and SIS scale to record their disease shame, chi-square analysis showed that SIS scores and negatively correlated with social support in patients with feeling (correlation coefficient is 0.60), showed that the lower the perceived social support, patients with the disease the more shame. An academic study [28] evaluated 135 patients with different types of preventive enterostomy by PSSS and other scales and found that self-efficacy rather than social support affected the quality of life of patients with preventive enterostomy, indicating that patients with preventive enterostomy had a lower need for social support, which was opposite to those with permanent enterostomy. It suggests that there is a certain difference in social isolation between prophylactic and permanent enterostomy patients.

#### 3.2.3. The Stoma Self-Efficacy Scale (SSES)

Due to the shortage of medical resources, enterostomy patients often have to be discharged from the hospital as soon as possible one week after the operation, and the lack of knowledge of self-care and perception of self-management of ostomy forces their quality of life to decline sharply [28], thus aggravating the social isolation of patients. Effective and regular ostomy nursing can help improve patients' sense of self-efficacy and has high application value.

The SSES was prepared by Bekkers et al. [29] and used to evaluate the self-efficacy of patients with ostomy. Likert 5-point scoring method was used to add points and sum. The higher the score, the better the self-efficacy of patients. The scale contains two dimensions (ostomy care self-efficacy and social function self-efficacy) and 29 items, among which 6 items are independent of the two dimensions, including ostomy self-efficacy and sexual efficacy [30]. Cronbach's *α* coefficients of the two dimensions are 0.94 and 0.95, respectively, explaining 61% of the total variation. Yan et al. [31] evaluated the self-efficacy of 74 colostomy patients 1 month after discharge and 3 months after discharge, the results showed that the overall level of self-efficacy of the patients was high, and the quality of life of the patients was high due to the average length of colostomy nursing within 1 month after discharge. It was suggested that the evaluation results of the SSES could provide transitional nursing measures for the patients with enterostomy and help them reduce the sense of social isolation such as self-esteem and frustration [32]. Knowles et al. [33] showed that self-efficacy is often manifested in the medium of disease cognition and disease response, which is particularly closely related to the mental health of patients. The fit index of self-efficacy evaluated by the SSES of patients with ostomy has high adaptability and strong correlation, which is one of the effective tools to understand the stigma of patients with ostomy. However, the self-efficacy assessment tool for distinguishing permanent and preventive enterostomy patients still needs to be revised and validated.

#### 3.2.4. Ostomy Adjustment Inventory (OAI)

OAI is an important tool used to assess the level of social psychological adaptation of patients with ostomy. Suffixes are added according to the different number of items to distinguish the scale versions. The first version is OAI-23 of Simmons et al., which was deleted and revised by Xu Qin et al. in 2010 to OAI-20, using 5-point Likert scoring method. Cronbach's *α* coefficient of the total table is 0.869, with good reliability [34]. Oai-30 was developed by Li [35]. The scale contains four dimensions and 30 items, including negative emotion (13 items), body function (9 items), treatment compliance (5 items), and survival anxiety (4 items, one of which is not scored). The Cronbach's *α* coefficients of the total scale and the four dimensions were 0.915, 0.893, 0.850, 0.754, and 0.774, respectively, which were well applied in the evaluation of stoma adaptation of 207 patients with permanent enterostomy after discharge. The results suggest that OAI-30 can help plan nursing interventions to improve patient adaptation to ostomy and avoid social isolation.

Although each scale appears to be independent of each other, in clinical application, multiple scales are often combined to evaluate the sense of social isolation of enterostomy patients, in order to obtain more accurate and detailed theoretical results and help reduce the incidence of adverse medical outcomes. RHDS, as a safety prediction tool for patients before discharge, is the earliest psychological measurement tool that enterostomy patients are exposed to during discharge transition period and plays an important role in preventing and improving the sense of social isolation. The combined use of SIS, PSSS, SSES, and OAI can predict and distinguish the psychological state changes of patients with preventive and permanent enterostomy in many aspects, so as to further realize the formulation and implementation of nursing plans.

## 4. Influencing Factors of Social Isolation in Enterostomy Patients during Discharge Transition Period

### 4.1. Patient Reasons

#### 4.1.1. Age

Age is one of the effective factors to predict social isolation of enterostomy patients after discharge. Scholar Li [35] investigated and evaluated the stigma of 234 discharged enterostomy patients for two years and found that age was negatively correlated with the score of stigma of patients, among which the score of stigma of patients ≤ 50 years old was as high as 85 points. The score of stigma in patients ≥ 61 years old is as low as 52, which may be related to younger patients paying more attention to external image and frustrated self-esteem [36, 37]. Psychological care should be carried out quickly for younger patients to reduce their sense of social isolation. It is worth noting that although it is generally believed that young age is an important factor promoting social isolation of patients with enterostomy, no systematic discussion or research on social isolation (stigma, etc.) of patients with enterostomy at different ages has been published, and the boundary between “young age” and “old age” is still controversial, which needs further confirmation.

#### 4.1.2. The Change Degree of Self-Body Image of Patients

Since patients with enterostomy cannot control excretion autonomously, they need to wear an ostomy bag continuously for 24 hours to collect excreta. This change in external image often leads to a surge in psychological pressure of patients [38], which intensifies the internalized sense of shame, thus prompting patients to isolate themselves and ultimately lead to their social derailment.

Patients' conscious body image change refers to patients' self-perception of their external image after enterostomy. Ye et al. [4] evaluated and studied the stigma of 131 patients with permanent enterostomy during the transitional period of discharge, and the SIS scale showed that 88.5% and 95.4% patients had severe internalized sense of shame and social isolation, respectively. Multiple regression analysis proved that the degree of conscious body image change was closely related to internalized shame and social isolation. The fitting equation explained 72.1% of the total variation, indicating that the degree of body image change was one of the important influencing factors for patients to develop stigma and self-isolation. And it may be related to impaired self-esteem. A foreign study [39] showed that the self-perception affecting the external image change of enterostomy patients had no difference in different genders, but was related to the patient's age, work situation, occupation type, social status, and cultural background. Jayarajah and Samarasekera [40] evaluated the influencing factors of adaptation disorders to body image changes in 41 patients with enterostomy. Smaller age, body mass index (bmi) of 23 kg/m2 or less, the types of preventive colostomy, the colostomy complications incidence rate is high, the operation time<2 years, and patients with colostomy function not congruent factor is in the hospital transition changes in body image perception and produce one of the important indices for bad mood, body image change closely related to intestinal colostomy patients psychological adaptation, It is of certain clinical significance to adopt correct nursing methods to improve patients' psychological adaptability and prevent social isolation.

#### 4.1.3. The Patient Self-Efficacy

The cognition, coping, and nursing of enterostomy are the evaluation indexes of self-efficacy of enterostomy patients after discharge and also the important factors that affect patients' normal state of mind during discharge transition period. Studies [41] showed that the permanent colostomy care intestinal colostomy patient self-efficacy and social self-efficacy are directly proportional to the quality of life of the patients after discharge, which patient self-efficacy is higher, the social psychological adaptation, the better, the less negative emotion, prompt the high level of self-efficacy is to prevent permanent social isolation of intestinal colostomy patients effective protection factors. However, the difficulty of ostomy care and its impact on stigma greatly limit the improvement of patient self-efficacy. Bulkley et al. [42] found that 63% of 177 patients with enterostomy experienced significant care challenges from peristomal skin complications and pocket replacement. It is closely related to the fact that the patient has no marriage partner (no partner to seek help), suggesting that the patients with enterostomy during the transition period of discharge have low ostomy care and social self-efficacy, which are more likely to induce the increased self-perceived burden of patients, increase their negative emotions, and affect their mental health [43]. Therefore, low self-efficacy is one of the key influencing factors mediating social isolation of patients after discharge.

#### 4.1.4. Patients' Acceptance and Support of Colostomy Bag

The colostomy bag is an important tool for patients with enterostomy to save excreta. Patients will reject and dislike the use of colostomy bag due to changes in body image and other reasons, which is one of the main manifestations of patients with strong stigma. Mac Donald and Anderson [44] showed that more than half of 420 discharged enterostomy patients held a negative attitude towards the application of the bag and refused to disclose the stoma to their spouse (33% of patients), family members (90%), and relatives and friends (90%) for help, suggesting that the patients had deliberately concealed the behavior, or it was related to their self-esteem. In addition, the unpleasant smell, noise, and possible leakage of colostomy bag also lead to low level of support for bag-making [38], thus mediating self-isolation, stigma, and other social isolation of patients, which should be paid attention to.

#### 4.1.5. The Social Support Degree

Social support refers to the floorboard of the various support from individuals, including friends and family support; family support, medical support, etc., are permanent intestinal colostomy patients, one of the seven spiritual demand of the system; the multidimensional social support can help patients with increased confidence and a sense of security [45] treatment; it is very important to patients after discharge can rely on. Multiple evidences show that low level of social support is an important influencing factor leading to low level of discharge preparation [46], negative emotions and negative psychological qualities [47], and stigma [4], suggesting that social support level is closely related to social isolation of enterostomy patients.

Discharge transition is a long process, and discharge readiness, as the first line of defense, is affected by subjective support. Subjective support is considered to be an emotional experience in which individuals are supported, understood, and respected. A high level of subjective support can alleviate patients' bad emotions and improve their stoma self-care efficacy [46], thus avoiding patients facing the disease alone, providing them with spiritual support, and weakening the sense of existence of social isolation.

The negative emotion and psychological quality of enterostomy patients lead to the sense of social isolation, which is closely related to the low level of social support. On the contrary, a high level of social support will promote patients' social adaptation and help them integrate into the social environment. Yang et al. [48] analyzed the self-perception of 16 patients with permanent enterostomy and found that patients' social support expectation was negatively correlated with patients' emotional support difference, indicating that low social support level was an important reason for patients' inability to obtain emotional maintenance and seriously affected their mental health. Nam et al.'s [49] research shows that 100 cases of surgical duration of 6 months or more intestinal colostomy patients in medical staff and the support of family members showed significant psychological adapt to change, including the support of the medical staff every increase 1 unit, the patient's psychosocial adaptation corresponding increased 0.04 units, adaptation level in patients with in time. It is suggested that effective medical support at the early stage of discharge is an important means to help patients adapt to the ostomy and social environment, which may be related to the improvement of the level of ostomy nursing and the shortening of the ostomy nursing time. Interestingly, the improvement in the level of family support in this study resulted in a decline in the patients' psychosocial adjustment. The fundamental finding is that inappropriate family support (such as disagreements caused by family religious differences) does not have a positive impact on the patients and even leads to adverse outcomes.

The low level of social support can also lead to and aggravate the stigma of patients, which seriously threatens the safety of patients' lives. Min [50] in 143 cases of permanent intestinal colostomy patients such as social influence, social support rating scale to assess their disease shame and the relationship between social support, found that the low level of subjective support and support utilization degree is the main factor of the disease shame patients, resulting in a higher social exclusion, internalize shame, and social isolation, and it suggests that social support is negatively correlated with stigma. Hu et al. [51] found that 118 patients with permanent enterostomy showed good adaptation to social life within 6 months after receiving peer support education, patients' ability of self-care of stomostomy was improved, and negative emotions and stigma were significantly reduced, proving the role of social support in improving patients' psychology and behavior. It also suggests that medical staff, families, and third parties should strengthen support for patients with enterostomy to help improve their quality of life.

### 4.2. The Type of Stoma and Postoperative Time

According to the duration, the types of colostomy can be divided into preventive (temporary) and permanent. The appearance of permanent patients will remain with them for their whole life, and patients often show serious negative emotions, which is an important factor leading to their social isolation.

According to the duration, the types of colostomy can be divided into preventive (temporary) and permanent. The appearance of permanent patients will remain with them for their whole life, and patients often show serious negative emotions, which is an important factor leading to their social isolation.

Gao et al. [25] evaluated the stigma of 193 patients with different types of enterostomy and found that the social isolation, social exclusion, and internalized shame of patients with permanent enterostomy were higher than those with preventive enterostomy, which may be related to the inability of patients with permanent enterostomy to recover their excretion function. Wang et al. [52] found that the social self-efficacy of patients with permanent enterostomy was significantly higher than that of patients with preventive enterostomy, which may be related to the higher demand for self-care of permanent enterostomy patients. In addition, along with the extension of time, postoperative two types of intestinal colostomy patients shame presents the downward trend, the disease is closely related to the level of social support [50], that transition period to give the correct discharge from hospital patients who are social support and improve the utilization efficiency of support to prevent social isolation, it is of great significance in the improve patients psychological status.

At present, there are few studies on inducing social isolation in patients with different types of ostomy and postoperative time during the transition period of discharge from hospital, which limits the real-time monitoring of patients' psychological state by medical institutions and may establish a channel of omission of social isolation supervision, thus affecting the quality of life of patients. In fact, although big probability to preventive intestinal colostomy patients recovered, but the patient worries too much or blind positive so it is easy to make it get lost after hospital discharge, excessive anxiety, or result in severe patients with negative emotions or suicidal behavior, and blind optimism will encourage patients to ignore the colostomy complications prevention and care in addition, focus too much on intestinal colostomy patients may also lead to permanent preventive intestinal colostomy patients psychological discontent, refused to communicate with family, the nurse, and the development of social isolation, these no detailed reports in the literature, further study of colostomy type, colostomy postoperative time these two factors make a thorough study, discharge guidance for clinical patients.

## 5. Conclusions and Prospects

With the development of medical technology, enterostomy has played a great role in the treatment of colorectal cancer and other diseases, providing reliable and efficient assistance to cancer victims at all ages. However, patients undergoing surgery are difficult to accept the change of body image. In the process of transition from hospital to social life, they often have serious negative emotions or social isolation, which affects their quality of life. At present, RHDS, SIS, PSSS, SSES, OAI, and other scales are mostly used in clinic to help monitor patients' mental health. These scales can evaluate patients' social exclusion, internalized shame, disease shame, and other types of social isolation and have good reliability and validity. When used in combination, they can detect the degree of social isolation at discharge and provide discharge guidance for patients. At the same time, patients can be followed up after discharge, and their psychosocial adaptation can be evaluated regularly, so as to achieve the goal of social isolation management. It can be determined that the influencing factors such as age, patients' conscious body image change, and patients' self-efficacy are closely related to the sense of social isolation in the transition period of discharge. One-to-one high-quality nursing has high application value in preventing adverse medical outcomes.

However, there are still some limitations in the existing research. Although the term social isolation has a development history of decades, the academic circles have not standardized its definition and interpretation. Whether social isolation is feeling or behavior is still an ambiguous problem, which makes it impossible to further understand the specific relationship between enterostomy patients and social isolation. Due to the limited medical resources, patients with enterostomy often begin to learn self-care of stoma and leave the hospital in a hurry about 1 week after operation. Although detailed and thorough research has been carried out on the mental health of patients after discharge, no research has focused on the changes of patients' social isolation in a complete discharge transition period. Finally, considering the long duration of stoma in patients with permanent enterostomy, there may be a misunderstanding in clinic, that is, the duration of stoma is directly proportional to the social isolation of patients, thus ignoring the mental health of patients with preventive enterostomy. In fact, patients with prophylactic enterostomy may need more social support and care than patients with permanent enterostomy, which may be a major reason to explain the high mortality of patients with prophylactic enterostomy.

At present, considerable progress has been made in the study of social isolation in patients with enterostomy during discharge transition period, and further research is urgently needed to explain and prove the above problems.

## Figures and Tables

**Figure 1:** The assessment of stigma.

## Data Availability

No data were used to support this study.
